This article has been retracted.

# *Vitis vinifera* L. Flavones Regulate Hippocampal Neurons via Autophagy in APP/PS1 Alzheimer Model Mice

**DOI:** 10.1155/2022/8554184

**Published:** 2022-09-01

**Authors:** Peng Zhang, Znafuguli Maimaiti, Gulixiati Aili, Fang Yuan, Hui Xiao

**Affiliations:** ^1^College of Public Health, Xinjiang Medical University, Urumqi, Xinjiang, China; ^2^College of Basic Medical, Xinjiang Medical University, Urumqi, Xinjiang, China

## Abstract

**Background:**

Alzheimer's disease (AD) is a neurodegenerative disease and our current treatment approach can only delay its course rather than cure it completely. Flavones from *Vitis vinifera* L. have been reported to promote synaptic plasticity and indirectly affect the expression of cholinergic neurotransmitters in a rat model of Alzheimer's disease.

**Objective:**

The aim of the study is to explore the effect of *Vitis vinifera* L. in APP/PS1 Alzheimer model mice.

**Methods:**

APP/PS1 AD mice were used as the research subjects, and the mice were divided into a model group, donepezil group, VTF low-dose group, VTF medium-dose group, and VTF high-dose group. C57BL/6 mice served as a control group. The autophagosomes were observed by a transmission electron microscope, and the expressions of LC3I, LC3IIand Beclin-1 were determined by Western blotting. The results of qRT-PCR are consistent with Western blotting.

**Results:**

VTF can exert a positive regulatory effect on AD mice by inhibiting autophagy.

**Conclusion:**

Our study supports that intragastrically administration of VTF is effective and operable in Alzheimer's disease mice, and that inhibition of excessive autophagy may be one of the potential reasons why VTF exerts a therapeutic effect on AD.

## 1. Introduction

Alzheimer's disease is a neurodegenerative disease that affects the elderly and is the most common cause of dementia in the elderly population [1]. The pathological hallmarks and typical symptoms of AD are the accumulation of senile plaques, neurofibrillary tangles, and progressive loss of memory [2–6]. However, the specific pathogenesis and causes of AD are still unclear. Currently, the scholars generally believe that it may be related to the environment, genetics, and aging. Conventional drugs in clinical practice at present, such as cholinesterase inhibitors and glutamate receptor antagonists, can only alleviate the disease process but cannot completely cure the disease [1, 7]. Therefore, exploring effective treatment strategies for AD is still an urgent problem to be solved in the scientific community.

Autophagy plays a crucial role in the development of many neurodegenerative diseases, and autophagy is considered to be a double-edged sword [8, 9]. Interestingly, most of our current scientific research on AD agrees that autophagy is beneficial in AD, and it might initiate self-protection through removing excessive intracellular peptide deposits and damaged organelles [10–15]. Beclin-1 is regarded as a marker protein of autophagosome formation and inhibiting the expression of beclin1 increases the deposition of A*β* in AD animal/cell models [16–18]. However, in some cases, hyperactivated autophagy has a negative effect on neuron survival. Therefore, inhibition of excessive autophagy may be an effective target for the treatment of AD.

Eating flavonoid-rich plants and fruits can repair damaged neurons [19]. *Vitis vinifera* L. flavones (VTF) is a flavonoid extracted from grapes. Recent studies have reported that VTF can promote synaptic plasticity, affect the expression of cholinergic neurotransmitters, and improve the learning and memory abilities in AD model rats [20]. However, it is unclear whether VTF can prevent hippocampal neurons damage through inhibiting autophagy. In this study, the changes of autophagy-related protein expression in the brain tissues were analyzed by qRT-PCR and western blotting. Our work revealed that the mechanism by which VTF exerts neuroprotective effects in AD models may be related to the suppression of excessive autophagy.

## 2. Materials and Methods

### 2.1. Animals

We purchased 6-month-old APP/PS-1 double-transgenic male mice (body weight (30 ± 10) g) from Promoter Biotechnology Co., Ltd. (Beijing, China) and used C57BL/6 mice as controls. A total of 90 mouse were selected, 15 in each group. Mice were housed under specific pathogen-free conditions, the environmental parameters were temperature 23 ± 2°C, humidity 60 ± 5%. The animal room where the mice were housed performed a 12 h light/12 h dark cycle, and the mice were given sufficient food, water and living space. All of the experiments followed the ethical guidelines of Xinjiang Medical University (Ethical approval number: IACUC-20210507-07.).

### 2.2. Preparation of Flavones from *Vitis vinifera* L

We added 95% ethanol to *V. vinifera* L. for extraction, then concentrated the extract into paste and mixed with water to form a suspension. AB-8 macroporous resin were used to elute and purify. Finally, the freeze-dried brown-yellow powder is VTF.

### 2.3. Animal Grouping and Drug Administration

We placed the experimental mice in the SPF laboratory and then administered the gavage after 1 week of adaptive feeding. 6-Month-old APP/PS1 AD mice were randomly divided into a model group and treatment group. The treatment group including a donepezil group (positive control), VTF low-dose group (70 mg/kg), a VTF medium-dose group (210 mg/kg), and a VTF high-dose group (420 mg/kg). The wild-type C57BL/6 male mice were taken as the control group, there are 6 groups in total. The model group were given the same concentration of CMC-Na solution (1.0 ml/100 g). All of the mice were intragastrically administered once a day (1.0 ml/100 g) for 8 weeks. Double blind method is adopted to avoid subjective influence. Mouse in normal control group were given distilled water by gavage; The positive control group was given donepezil solution (donepezil powder dissolve in distilled water and shake well with 0.5 mg/kg) by gavage.

### 2.4. Western Blot

We collected mice hippocampus tissues and extracted the protein solution. We then tested the protein concentration in each sample with BCA kit. We separated the protein through SDS-PAGE and transferred it onto PVDF membranes. After blocking the excess binding sites on the membrane with nonfat dry milk, the PVDF membranes were incubated at 4°C with the following antibodies for one night (primary antibodies): LC3-I (1: 500, Abcam, LC3-II (1: 500, Abcam), Beclin-1 (1: 500, Abcam) and GAPDH (1: 500, Abcam). The PVDF membranes were washed with PBS supplemented with 0.1% Tween 20 and then incubated with the corresponding secondary antibody for 1 h at room temperature. The membranes were visualized using an LAS-4000 chemiluminescence detection system. We used Image J software to quantify the band densities.

### 2.5. Quantitative Reverse Transcription-Polymerase Chain Reaction (qRT-PCR)

According to the kit instructions (ThermoFisher Scientific., Carlsbad, United States), total RNA from hippocampus tissues was extracted and reverse-transcribed into cDNA. After adding the fluorescent dye, the quantitative real-time PCR was performed using quantitative PCR (Applied Biosystems, CA, United States) with corresponding primers (Table 1). The levels of mRNA were normalized in relevance to GAPDH.

### 2.6. Transmission Electron Microscopy

Brain tissues were fixed with 6% glutaraldehyde and cut into slices, and then we stained these slices with lead. We observed and photographed autophagosomes in the mice hippocampus using transmission electron microscopy.

### 2.7. Statistical Analysis

We used SPSS software (version 20.0) and GraphPad Prism 6 software (version 4.0) to performed statistical analyses and data are presented as mean ± SEM. The data of western blot and qRT-PCR were analyzed by one-way ANOVA followed by the *post hoc* Bonferroni multiple comparison test. *P* < 0.05 was considered statistically significant.

## 3. Results

### 3.1. *Vitis vinifera* L. Flavones Can Inhibit Excessive Autophagy in Hippocampus

The autophagy-related proteins LC3-I, LC3-II, and Beclin-1 were identified. Western blot results showed that the protein expression of Beclin-1 in the model group was significantly higher than that in the treatment group (Figure 1. *P* < 0.05), and in the treatment group, the expression level of Beclin-1 was negatively correlated with the dose of VTF. We speculate that the significantly decreased expression of beclin1 after treatment was related to the repression of autophagy. In addition, we tested the change trend of LC3-II/LC3-I, our result indicated that the excessive autophagy in hippocampus was inhibited, which further confirmed our previous conjecture.

To further verify the role of VTF in regulating autophagy from the gene level, we extracted total RNA from mice hippocampus and performed RT-qPCR. The mRNA levels of LC3 and Beclin-1 in the hippocampus of the model group were much higher than those of the treatment group, and the decrease of LC3 and Beclin-1 in the treatment group were VTF concentration-dependent, and the difference among the groups was statistically significant (*P* < 0.01, Figure 2). The gene expression trend of p62 is consistent with Beclin-1 and LC3; we speculate that this may be because the mechanism by which VTF exert the positive effects through inhibiting excessive accumulation of autophagy. Our results demonstrate that VTF can repress the expression of pro-autophagy-related proteins in the hippocampus. These results confirm those of the Western blot.

The autophagosomes were detected in the hippocampus using TEM in a ×4.0 k field of view (Figure 3). Compared with the model group, the number of autophagosomes in the treatment group grow in number with the decreasing dose of VTF. In fact, the model group has the highest number of autophagosomes. Therefore, the researchers speculated that VTF could exert its positive effects by suppression autophagy in the hippocampus.

Based on the above experimental results, we believe that *Vitis vinifera* L. Flavones. can inhibit excessive autophagy in hippocampus.

## 4. Discussion

Flavonoids are polyphenolic compounds that are widely present in plants and can be successfully extracted from tea, cocoa, and wine [21–23]. Emerging evidence suggests that flavonoids can act as oxygen free radical scavengers and antioxidants [24, 25]. Flavonoids can smoothly cross the blood-brain barrier (BBB) in neurological diseases [26], it can exert neuroprotective and anti-inflammatory effects in the central nervous system and improve learning and memory in memory-impaired mice [27–30]. Studies have shown that a variety of flavonoids may have positive therapeutic effects on AD. Vepsäläinen et al. and colleagues fed APP/PS1 mice with anthocyanin-enriched bilberry and blackcurrant extracts, they found that it alleviated spatial working memory deficits and altered amyloid precursor protein (APP) processing [31]. In addition, Nobiletin, a citrus flavonoid, was found to improve memory impairment and Abeta pathology in a transgenic mice model of Alzheimer's disease [32]. Flavonoids can also reduce amyloid beta production in AD by mediating presenilin-1 phosphorylation [33]. In general, flavonoids are currently very promising drugs for the treatment of AD.

Previous studies have shown that VTF can promote synaptic plasticity and indirectly affect the expression of cholinergic neurotransmitters [20]. Our work attempts to explore the underlying mechanisms more deeply from the perspective of autophagy. We believe that this positive effect of VTF may be related to inhibiting excessive autophagy in Alzheimer's disease model mice.

The metabolism of A*β* and Tau is strongly associated with autophagy, regulating autophagy is regard as one of the most promising therapeutic strategies [34–37]. Under normal circumstances, activation or a certain degree of enhancement of autophagy can significantly eliminate A*β* deposition, promote Tau clearance, and alleviate neurodegeneration [34, 38, 39]. Some researchers added A*β*_1–42_ to SH-SY5Y cells and found that it can cause a certain cytotoxic effect on the cells. After administering rapamycin (an autophagy inducer), it can not only reduce the level of A*β*_1–42_ but also exert a protective effect in SH-SY5Y cells [40]. In the APP/PS1 AD mouse model, it was also found that activating autophagy could reduce senile plaques formed by A*β* deposition and alleviate memory and cognitive impairment in mice [14, 41–44]. In addition, the formation of autophagosomes is also often accompanied by a decrease in the content of phosphorylated Tau [45, 46]. However, there are also some research results supporting that autophagy does not always play a positive role in AD models. ATG7 is an essential protein for cellular degradation and recycling associated with autophagy. Some scholars have tried to cross the amyloid precursor protein (APP) transgenic mice with ATG7-selective knockout mice. It was found that A*β* secretion was inhibited due to the lack of autophagy, and it was surprising to find that the burden of extracellular A*β* protein was greatly reduced. [47, 48]. Both of these opposite results have been scientifically verified in a certain degree. Our team believes that the reason for this phenomenon may be because the two-sided nature of autophagy itself makes it play different effects in different situations. Maybe it is a good choice to bring the level of autophagy back to a balanced level.

A previous interesting study observed that VTF can enhance synaptic plasticity and improve cognitive impairment in AD model mice, which indicates that VTF has a great therapeutic potential in neurodegenerative diseases [20]. Our work attempts to build on the previous work to further investigate the reasons why VTF plays a positive role and its possible relationship with autophagy.

### 4.1. Limitation

“Autophagy” itself is a complex concept. We did not evaluate the change of autophagy flow nor did we conduct a control experiment to observe whether the positive effect of VTF can be reversed after using autophagy inhibitors. Relevant research will be further carried out in the future.

## 5. Conclusion

Based on the above research work, we believe that VTF can affect the pathological changes of Alzheimer's disease by inhibiting excessive autophagy. This discovery provides a new theoretical basis for the therapeutic prospects of VTF in the treatment of Alzheimer's disease.

## Figures and Tables

**Figure 1:** VTF administration inhibits excessive autophagy In AD models. Representative western blots and quantitation data of apoptosis-related proteins. (a) The levels of the apoptosis-related proteins are reported as the value normalized to GAPDH for each sample. (b–d) Compared to the model group, the mean percentage of beclin1, LC3-II, LC3-II/LC3-I was significantly decreased in the treatment group. Relative expression expressed as the mean ± SEM. ^#^The *p*-value was less than 0.01 compared with the control group. ^*∗*^The *p* value was less than 0.05 compared with the model group. ^*∗∗*^The *p* value was less than 0.01 compared with the model group.

**Figure 2:** Comparison of relative mRNA expression of autophagy-relate proteins in different groups. (a–c) Compared to the model group, the mean percentage of beclin1, LC3, P62 was significantly decreased in the treatment group. Relative expression expressed as the mean ± SEM. ^#^The *p*-value was less than 0.01 compared with the control group. ^*∗*^The *p* value was less than 0.05 compared with the model group. ^*∗∗*^The *p* value was less than 0.01 compared with the model group.

**Figure 3:** Electron microscopy-based detection of autophagosome in hippocampal neurons. Representative images of autophagosome in the six groups, the autophagosome was observed under an electron microscope at ×4.0 k magnification (bar = 500 nm). Compared with the model group, the number of autophagosomes in the treatment group grow in number with the decreasing dose of VTF. ^*∗*^The *p* value was less than 0.05 compared with the model group. ^*∗∗*^The *p* value was less than 0.01 compared with the model group.

**Table 1:** Primer sequence of q RT-PCR.

Gene	Primer	Sequence (5′-3′)	PCR products
Mus GAPDH	Forward	ATGGGTGTGAACCACGAGA	229bp
	Reverse	CAGGGATGATGTTCTGGGCA	

Mus Beclin-1	Forward	GATTGGACCAGGAGGAAG	160bp
	Reverse	AAGGTGGCATTGAAGACA	

Mus LC3	Forward	AATGCTAACCAAGCCTTCTTCCTCC	103bp
	Reverse	AGCCGTCTTCATCTCTCTCACTCTC	

Mus p62	Forward	CCTGAAGAATGTGGGGGAGAGTGTG	122bp
	Reverse	TGGAACTTTCTGGGGTAGTGGGTGT	

## Data Availability

The data used to support the findings of this study are available from the corresponding author upon request.
